# A Deep Learning-Based Classification Method for Different Frequency EEG Data

**DOI:** 10.1155/2021/1972662

**Published:** 2021-10-21

**Authors:** Tingxi Wen, Yu Du, Ting Pan, Chuanbo Huang, Zhongnan Zhang

**Affiliations:** ^1^College of Engineering, Huaqiao University, Quanzhou 362021, China; ^2^Postdoctoral Workstation of Linewell Software Company Limited, Quanzhou 362000, China; ^3^School of Informatics, Xiamen University, Xiamen, China

## Abstract

In recent years, the research on electroencephalography (EEG) has focused on the feature extraction of EEG signals. The development of convenient and simple EEG acquisition devices has produced a variety of EEG signal sources and the diversity of the EEG data. Thus, the adaptability of EEG classification methods has become significant. This study proposed a deep network model for autonomous learning and classification of EEG signals, which could self-adaptively classify EEG signals with different sampling frequencies and lengths. The artificial design feature extraction methods could not obtain stable classification results when analyzing EEG data with different sampling frequencies. However, the proposed depth network model showed considerably better universality and classification accuracy, particularly for EEG signals with short length, which was validated by two datasets.

## 1. Introduction

Epilepsy is characterized by recurrent seizures caused by the abnormal discharge of brain neurons, which often bring physical and psychological harm to patients. Approximately 50 million epilepsy patients have been documented globally, and epilepsy has become one of the most common nervous system diseases endangering human health worldwide. Brain wave is a synaptic postsynaptic potential generated by numerous neurons when the brain is active. It can record brain wave changes during brain activity and reflect the electrophysiological activities of the cerebral cortex or scalp surface of brain neurons [1]. Accordingly, brain wave analysis has become an effective and important method for the study of epilepsy.

Since the 1980s, scholars have been conducting research on epilepsy based on electroencephalography (EEG), among which the identification of epilepsy by analyzing EEG data is one of the important research contents [2]. With the development of computer science and technology, numerous studies have focused on the classification of features extracted from EEG signals by using a computer classification model [3, 4]. Such a research often follows the following steps: EEG data acquisition and prepossessing, feature extraction, classification model training, and data prediction. Feature extraction from EEG data is one of the most important steps. Numerous methods are used to extract EEG features, including time-domain, frequency-domain, and time-frequency analyses and chaotic features [5–7]. Moreover, some studies have combined or redesigned these methods to obtain new features, thereby eventually achieving good classification results [8–10].

With the development of science and technology, the accuracy of medical EEG acquisition equipment has been improved. In addition, some portable EEG acquisition equipment has been developed. For example, emotive has been widely used in brain-computer interface [11–13] because it is lightweight and inexpensive and has similar performance to medical equipment. However, although a variety of medical devices or portable EEG acquisition devices produce numerous EEG data that can be used for epilepsy research, the different data sources result in a lack of uniform data formats, such as different sampling frequencies, different signal lengths, and different sampling channels. The inconsistency of data specifications often affects the features obtained by traditional feature extraction methods. This situation raises a question on how to improve the ability of classification methods to adapt to new data. Hence, the universality of classification methods should be improved, while ensuring the enhanced detection and recognition of EEG data.

At present, in-depth learning technology is a popular research area. Given this technology's autonomous learning characteristics from data, it can directly skip the manual design features and extraction process in the traditional methods, avoid the difficulties of manual design features in traditional methods, and manually adjust numerous parameters. In-depth learning technology can accomplish numerous tasks that are difficult to complete in the traditional methods [14]. Some researchers have studied EEG via a deep network [15]. Tabar and Halici [16] converted one-dimensional (1D) brain waves into two-dimensional (2D) image data through short-time Fourier transform and accessed the deep network for classification. Bashivan et al. [17] converted the frequency bands extracted from brain waves into topographical maps (2D images) through spectral power and classified the images into depth networks. Hosseini et al. [18] used an in-depth learning method based on a cloud platform to propose a solution for epilepsy prevention and control. Xun et al. [19] and Masci et al. [20] proposed a coding method for epileptic EEG signals based on the deep network. However, the majority of these studies have focused on regular data, such as the same frequency and same length of the sample data. In the feature design aspect, these studies have converted 1D EEG data into 2D image data in advance and classified the features via the deep network. The current study constructed a classification model based on the deep convolution network to automatically learn the characteristics of EEG and adapt to the EEG data of different sampling frequencies and lengths. Our method (including network model and training method) can considerably identify different forms of EEG data.

The remainder of this paper is organized as follows.  Section 2 first simulates the EEG data with different frequencies. Thereafter, we classify the data with existing manual feature design classification methods and indicate their disadvantages compared with our model.  Section 3 provides details of our proposed network model, training methods, and data processing methods.  Section 4 compares our model with existing methods and discusses the advantages of our model.  Section 5 presents the summary.

## 2. Experimental Result

This section first describes two open datasets and classifies and compares the EEG data at different sampling frequencies using an artificial design feature method and deep network autonomous feature learning method.

### 2.1. Data Description and Data Synthesis

#### 2.1.1. Dataset 1

The first dataset comes from the dataset published by Andrzejak et al. [21]. This dataset consists of five subsets (represented as A to E). Each subset contains 100 EEG signals of 23.6 sec in length, and the sampling frequency is 173.6 Hz. The data include records of healthy and epileptic patients. Among them, there were two subsets of EEG recorded during epileptic seizures, which had 200 samples, and one set of EEG records in the seizure period had 100 samples.  Figure 1 shows two types of signals in epilepsy patients during nonepilepsy and epilepsy. They are classified as F and S, respectively. Among them, 200 samples are classified as F and 100 samples are classified as S. Class F is labeled as a nonepileptic seizure EEG signal, while class S is a seizure signal.

#### 2.1.2. Dataset 2

The second dataset was collected by Boston Children's Hospital [22]. EEG signals are obtained by measuring electrical activity in the brain by connecting multiple electrodes to a patient's scalp. Data length is approximately from half an hour to one hour, including epileptic seizure and nonepileptic data. The sampling frequency of each data sample is 256 Hz, which contains 23–25 channels, and the sample length is approximately 921600. The dataset has 24 subjects. The first 10 subjects are selected for experiment. Each channel in the sample has a name; for example, the first channel was named FP1-F7 (see Figure 2). We selected one of the 23 channels for our study. When epilepsy occurs, the EEG signal will fluctuate substantially, resulting in an increase in the signal variance. We make channel selection based on variance [23]. The method is as follows. We calculate the variance of each channel in each sample, with each sample having a channel with the largest variance, and derive the statistics on these channels thereafter with the largest variance in the sample. The “FT9-FT10” channel has the highest number of occurrences, thereby leading us to choose this channel. A total of 200 EEG samples of epileptic seizures and 200 nonepileptic seizures were randomly intercepted on the FT9-FT10 channel. The length of each signal sample was 4096 (or 16 sec). Class F remains to be labeled as a nonepileptic seizure EEG signal in dataset 2, while class S is a seizure signal.

The signal is a cortical signal, the signal on the left side of the black line is no epilepsy, and the signal on the right side of the black line is epilepsy, as shown in Figure 2.

The two datasets are the most widely used in the current research on epilepsy data classification and detection. Given that the sampling frequency of signals in the two datasets is fixed, we use the signal processing library in SciPy [24] to obtain additional EEG data with different sampling frequencies, particularly to resample the existing data and obtain a new sampling frequency dataset thereafter. For example, the sampling frequency of the original dataset 1 is 173.61 Hz, and the original dataset is resampled at 163.61, 153.61, 143.61, 133.61, 123.61, 113.61, and 103.61 Hz (decreasing at 10 Hz). In this example, 1-0 represents the original 173.61 Hz data and 1-1 represents the 163.61 Hz data. By analogy, the resampled new dataset is shown in Table 1.  Table 2 shows that for the resampling of data 2, the sampling frequency of the original dataset 2 is 256 Hz. In this example, the original dataset 2 is resampled at 236, 216, 196, 176, 156, 136, and 116 Hz (decreasing at 20 Hz). Hence, new datasets can be obtained, in which 2-0 still represents data of the original dataset 2.

### 2.2. Classification Results Based on the Artificial Design Feature Extraction Method

Features or design new features should be selected for classification based on the artificial design feature extraction method. The current study selects the feature extraction methods [25–27], which have a good classification effect in the existing research, including integral absolute value, root mean square, waveform length, sample entropy, Lee's index, Hurst index, DFA index, and multifractal feature. After feature extraction, several common classifiers are selected from the scikit-learn library [28], including *k*-nearest neighbor (*k*-NN), linear classifier (LDA), support vector machine (SVM), decision tree (DT), multilayer perceptron (MLP), and Gaussian naive Bayes (GNB). These classification algorithms adopt self-contained parameters in the library. Tables 3 and 4 use the aforementioned features and classifiers to classify datasets 1-0 and 2-0, respectively. The table shows the results of the 3-, 5-, and 10-fold cross-validations. The last column of AVG is the average classification accuracy of each classifier. SVM, which is the commonly used classifier, achieves good classification accuracy and validates the effectiveness of the feature extraction methods.

Tables 5 and 6 show the accuracy of the 5-fold classification of datasets by various classifiers.

Table 5 shows that under different sampling frequencies, traditional classification methods based on artificial design feature have different classification results in different classifiers. For example, the classification results of SVM should be optimized to GNB. When sampling frequency decreases, classification accuracy fluctuates. For example, the classification accuracy of *k*-NN decreases, and those of LDA and SVM change substantially.  Table 6 shows that the average accuracy of the last column is higher than that of Table 5. This result indicates that the classification method based on artificial design features can achieve superior classification results in datasets 2-0 to 2-7. However, the classification accuracy of data with different sampling frequencies continues to fluctuate significantly.  Figure 3 shows the average classification accuracy of two datasets based on artificial design features at different sampling frequencies. The classification results of datasets 1-0 to 1-7 are not ideal, while datasets 2-0 to 2-7 have better classification results. These synthesizations show that the method based on artificial design features depends on the selection of classifiers. Moreover, this method's characteristics are sensitive to the data of different sampling frequencies, which substantially reduces the applicability of the method.

### 2.3. Classification Results Based on the Convolutional Neural Network

This section presents the classification results of the self-learning feature method based on the convolutional neural network (CNN) for the preceding datasets. Tables 7 and 8 categorize the two datasets at different sampling frequencies. A comparison of Tables 5 and 6 indicates that our model has more stable classification results and better classification accuracy.

The results of training and testing for the same sampling frequency data are listed in Tables 1to 6. Whether or not these methods are effective in the case of mixing various frequency data needs further analysis. Moreover, whether or not a classification model can train the datasets of existing sampling frequencies and effectively predict the data of new sampling frequencies should be further discussed. For example, the model is trained with the 173.61 Hz and 163.61 Hz data to predict the type of the 153.61 Hz data. Given these problems, the third part of this paper explains the solutions and further discusses and analyzes these problems in the fourth part.

## 3. Methodology

This section first describes the model structure based on CNN and the training methods for different length sample data.

### 3.1. Classification Model Based on CNN

Numerous methods of feature extraction are based on artificial design. However, when the data changes, the classification effect based on the general feature extraction method is not stable. In this study, the classification model based on CNN can independently learn and classify data features, including the two steps of feature extraction and classification (see Figure 4). It attempts to obtain good and stable classification results when facing different sampling frequencies or different lengths of the sample data.

The left side is a classification process based on artificial design features, which requires two steps. The right side is to input data into the network model and output the classification results directly, as shown in Figure 4.

CNN is a feedforward neural network that improves the classification ability of patterns by posterior probability. The network mainly includes convolutional, pooling, fully connected, and softmax layers. The convolution layer convolutes the input signal data through different convolution kernels to obtain the feature map (i.e., number of convolution kernels equals the number of feature maps). The pooling layer is the process of downsampling the feature map obtained from the convolution operation of the upper layer. The network often increases the network depth by iterating the convolutional and pooling layers. Meanwhile, the fully connected layer connects all feature maps from the upper layer to the hidden layer of a common neural network and eventually outputs the classification results through the softmax layer. This study proposes a multilayer network with cubic iterative convolutional and pooling layers, fully connected layer, and softmax layer to classify EEG data (hereinafter referred to as CNN-E). The model classifies the one-dimensional EEG data of a single channel and makes the input sample data *X*. The convolutional layer is equivalent to the feature extractor. This layer uses multiple convolution kernels to convolute *x* and obtains several feature maps that can keep the main components of the input signal. The convolution calculation formula is as follows:

(1) $$\begin{array}{c} f_{n}^{k}=g_{k}\left(\underset{\forall m}{\sum }\left(f_{m}^{k-1}*w_{m,n}^{k}\right)+b_{n}^{k}\right), \end{array}$$

where *f*_*n*_^*k*^ represents the feature map of layer *k*, *f*_*m*_^*k*−1^ is the feature map of the upper layer, *w*_*m*,*n*_^*k*^ represents the convolution kernels of the *m*th feature map of layer *k* − 1 to the *n*th feature map of layer *k*, *b*_*n*_^*k*^ is the neuron bias, and *g*_*k*_(·) is the activation function. When *k* = 1, that is, the first convolution operation on sample data, *f*_*m*_^*k*−1^ = *x* and *M* = 1, because only one feature map in the upper layer is *x* and *N* is the number of convolution kernels. Given that the input data *X* is one-dimensional, the feature map *f*_*n*_^*k*^ output by convolution operation is also one-dimensional. In this model, the pooling operation divides *f*_*n*_^*k*^ with length *l* into *J* regions of equal length without overlap, and each region has *i*/*j* elements and extracts the maximum value from each region. Hence, the size of the feature map can be reduced to a downsampling. In this way, the strongest features in each region can be selected, and the ability to distinguish the overall features of the model can be enhanced. After the pooling operation, *f*_*n*_^*k*^ changes from the original length *l* to *j*, where the maximum pooling operation is *p*_*k*_(*f*_*n*_^*k*−1^, *i*), and *i* = *l*/*j* is the reduction ratio of the feature map. Thereafter, the pooling operation is as follows:

(2) $$\begin{array}{c} s_{n}^{k}=p_{k}\left(f_{n}^{k-1},i\right). \end{array}$$

Each neuron in the fully connected layer connects to all neurons in the upper layer *f*_*n*_^*k*−1^. The output of all neurons in the upper layer *f*_*n*_^*k*−1^ is mapped to a dimension array *V* by reshape operation, and *V* is input to the fully connected layer. Thereafter, the fully connected layer can be expressed as follows:

(3) $$\begin{array}{c} c=g_{c}\left(v*w_{c}+b_{c}\right), \end{array}$$

where *w*_*c*_ and *b*_*c*_ are the weights and biases, respectively, of the fully connected layer and *c* is the output of the fully connected layer. Lastly, the final result is output via softmax, and the operation is as follows:

(4) $$\begin{array}{c} y=\text{softmax}\left(c\right). \end{array}$$

The classification result *y* is obtained.

Assuming that there are *N* training samples, *x*^(*i*)^ represents a sample labeled *l*^(*i*)^. Sample *x*^(*i*)^ is calculated by the model to obtain *y*^(*i*)^. Thereafter, cross-entropy is used as the loss function of the model. The formula is as follows:

(5) $$\begin{array}{c} \text{Loss}\left(x\right)=-\underset{i}{\sum }l^{\left(i\right)}\log\left(y^{\left(i\right)}\right). \end{array}$$

The loss function of the network model is optimized by the SGD [26] optimizer.

### 3.2. Model Training

Section 3.1 explained the basic structure and principle of the CNN-E model. This section further introduces the parameter setting and model training of the model.

Figure 5 shows the CNN-E frame diagram of the neural network model used in this research. Given that a sample signal is stored in an array, each small rectangle in the graph represents the elements of the signal, and numerous small rectangles constitute a sample signal. The length of the input sample signal is 4096. After the calculation of three convolution layers, the number of convolution kernels in the first, second, and third convolution calculations are 16, 32, and 64, respectively. After each downsampling, the signal length changed to half of the original length, and the number of neurons in the fully connected layer was 64. In the first convolution operation, the sigmoid function is used as the activation function, while the ReLU function is used as the other activation functions.

After determining the model, we input training samples to train the model. We know that the length of each sample in datasets 1-0 and 2-0 is 4096, and the length of the new frequency data obtained by resampling changes. The resampling method is operated using the Fourier resampling method in the signal processing toolkit of SciPy. In Figure 6(a), one sample in dataset 1-0 and four new samples (i.e., 1-1, 1-2, 1-3, and 1-4) generated by the sample at different sampling frequencies are presented. With the decrease in sampling frequency, the sample length becomes considerably short. However, the length of input data acceptable to the model is fixed. This study used the complementation method to cut a certain length of data from the head of the sample and supplement it to the tail. Thus, the length of the sample data reaches 4096. Figure 6(b) shows that the data in the red rectangle is replicated and supplemented to the blue rectangle. In this way, the model can be adapted to different length data. If the sample data is above 4096, then the 4096-length data is input into the model.

To enhance the universality of the model, there is no data preprocessing operation in data training. For example, the majority of the data in dataset 1 range from −500 to 500, and a small part of the data may be extended to −2000 to 2000 owing to abnormal or noise fluctuations. Thereafter, the sigmoid function used in the first convolution can reduce the impact of these abnormal data on model training.

Figure 6(a) is the new data generated by using different sampling frequencies for the original data, and Figure 6(b) is the sample data after completing the data in Figure 6(a).

## 4. Discussion

This section compares the classification results of the artificial design feature method and CNN-E model and different sampling frequencies.

### 4.1. Comparative and Characteristic Analyses of the Classification Results with the Same Frequency

Data were trained and classified at the same sampling frequency.  Figure 7 shows the classification accuracy of the two methods for two datasets. Among them, A represents the average classification result of the classification method based on artificial design features. B is the classification result of the current CNN-E model. In datasets 1-0 to 1-7, we find that the classification accuracy of the CNN-E model is above 0.95, which has a good classification effect. In datasets 2-0 to 2-7, the classification accuracy of only 2-0 and 2-2 is lower than that of the classification method based on artificial design features. The majority of the others are higher than those of the classification method based on artificial design features. Moreover, we find that for the two datasets, the classification accuracy tends to decline with a decreasing frequency of adoption. CNN-E continues to maintain relatively stable classification accuracy.

A is a classification method based on artificial design features, and B is a classification method based on CNN-E, as shown in Figure 7.

Figure 8 shows the distribution of the F and S data features in datasets 1-0 and 1-7. Under different sampling frequencies, the calculated distribution of features is relatively different. For example, the two types of features are easy to distinguish in *f*_1_, the two types of features in *f*_6_ and *f*_11_ are nearly unchanged, and the feature *f*_5_ becomes difficult to distinguish. These aspects reflect that the artificial design feature method is considerably dependent on the actual data signal. When the sampling frequency changes, the feature distribution also changes. This situation is also the reason why the classification accuracy decreases with a decrease in sampling frequency in the preceding experiments. From the classification results of datasets 2-0 to 2-7 in Figure 3, the artificial design feature method remains effective. First, the majority of the features (12) are used. Second, Figure 7 shows that these features change regularly at different sampling frequencies. Lastly, these features are selected from the existing features with good experimental results. However, the performance of these features in datasets 1-0 to 1-7 is poor, which also shows that the classification methods based on artificial design feature extraction have considerable differences in the performance of different datasets. However, the features obtained by CNN-E have profound meanings and local features. Although these deep features are difficult to visualize, they have good adaptability, as shown in Figure 7.

In the previous section, the classification method based on artificial design feature design and the classification results of CNN-E at the same sampling frequency are analyzed. This section uses the classification results of different sampling frequency data to show the universality of the CNN-E model.  Figure 9 shows that some characteristic distributions of the sample data will change at different sampling frequencies. Given that the data resampling method is based on the Fourier resampling method, the characteristic changes in the frequency domain are relatively small.  Figure 9 shows the spectrum of samples at different sampling frequencies.  Figure 9(a) lists the spectrum obtained by applying different sampling frequencies to the same sample. This series of spectrum is nearly identical in the blue rectangular frame. To ensure that the model can be adapted to data of different lengths, the length of input samples is supplemented by the complementary method (see Figure 6). The spectrum also changes after completing the sample data of different sampling frequencies. For example, Figure 9(b) shows that with the change of sampling frequency, the spectrum of the new sample is increasingly different from that of the original sample.

Figure 9(a) is listed as the spectrum of samples at different sampling frequencies, and Figure 9(b) is listed as the spectrum of samples after the complementation method.

Figure 10 shows that the classification results of the CNN-E model for different frequency sampled data are better than those of the traditional classification methods based on artificial design features (e.g., *k*-NN, LAD, and SVM). Although there are considerable differences in the spectral characteristics of samples when the input sample signal is supplemented, the CNN-E model can extract deep features and reduce the feature dimension of the samples. Hence, the model achieves a good classification effect.

### 4.2. Nonequal Length Sample Testing

In practical application, the EEG classification model faces different sampling frequency data and can also process different lengths of signal data. However, numerous artificial design features have constraints on data length when extracting features. For example, when data length is only one second or the sampling frequency is not high, meaningful time-domain, frequency-domain, or nondynamic features cannot be extracted. Previous classification studies are mostly based on time windows. All samples are divided into new sample sets according to a certain length of time windows, and training and test sets are divided thereafter for training and testing, respectively, the model. Given that the proposed model can be adapted to different lengths of the sample data, we use the experiments in the previous section as bases in utilizing different lengths of time windows to segment the sample data without overlap. The window length is 1 sec, 2 seconds to the signal length. If the sample length of dataset 1-0 is 23.6 sec, then its maximum window length is 23 sec. The sample length of dataset 2 is 16 sec, and its maximum window length is 16 sec.  Table 9 shows that datasets 1-0 and 1-1 are divided into different time lengths of 1 to 5 sec, respectively, and the changes of the sample length and sample number are obtained.

Figure 11 shows the classification accuracy of different datasets divided by different time lengths based on the CNN-E classification model. From the graph, the model proposed in this research achieves a good classification effect (i.e., amount of data in 1 sec can obtain a high classification accuracy) and has high timeliness on the premise of ensuring high accuracy.

## 5. Conclusion

In real life, there are diverse types of EEG signals. The current research on EEG classification has focused on classification accuracy, but the universality of the methods has seldom been discussed. To solve the problem, this study constructed a CNN-E classification model based on CNN. The model could be applied to classify EEG signals with different sampling frequencies and could be adapted to signals of different lengths. This study also analyzed the possible problems in the classification of EEG signals with different sampling frequencies by the traditional feature extraction-based classification method. Our results showed that the traditional method has relied heavily on the design of the feature extraction method, and there were difficulties in feature design and selection. Moreover, the classification accuracy fluctuated substantially for EEG data with different sampling frequencies. These feature extraction methods had length constraints when processing samples with short data length. However, the CNN-E model could independently learn the characteristics of the sample data and could be adapted to all types of data length because of the use of effective data completion methods. Our results showed that the CNN-E model performed well in the classification of EEG data at the same sampling frequency, at different sampling frequencies, and at different lengths.

Although we only used two different datasets to test the robustness of the CNN-E model, we would use additional datasets to validate the reliability of this model in the future. Moreover, the performance of the CNN-E model, particularly the visual expression of the features learned by the CNN network, needs further improvement.

## Figures and Tables

**Figure 1:** Signal samples of categories F and S in dataset 1.

**Figure 2:** Signal samples of dataset 2.

**Figure 3:** Generation of new datasets for the two original datasets and the average classification results of 3-, 5-, and 10-fold.

**Figure 4:** Process diagram of the artificial design features and network learning model.

**Figure 5:** CNN-E framework diagram of the neural network model.

**Figure 6:** Completion of sample data at different sampling frequencies.

**Figure 7:** Comparing the classification readiness of the two methods at the same sampling frequency.

**Figure 8:** Classification of the F and S features in dataset 1 in 1-0 and 1-7.

**Figure 9:** Spectrum of samples at different sampling frequencies.

**Figure 10:** Tests of the classification accuracy of the current frequency data using other sampling frequency trainings.

**Figure 11:** Secondary classification accuracy of samples based on the CNN classification model.

**Table 1:** List of datasets obtained after resampling for dataset 1.

Dataset name	Sample frequency (Hz)	Sample length	Time length (s)
1-0	173.61	4096	23.6
1-1	163.61	3861	23.6
1-2	153.61	3625	23.6
1-3	143.61	3153	23.6
1-4	133.61	3389	23.6
1-5	123.61	2917	23.6
1-6	113.61	2681	23.6
1-7	103.61	2445	23.6

**Table 2:** List of datasets after resampling for dataset 2.

Dataset name	Sample frequency (Hz)	Sample length	Time length (s)
2-0	256	4096	16
2-1	236	3776	16
2-2	216	3616	16
2-3	196	3136	16
2-4	176	2816	16
2-5	156	2496	16
2-6	136	2176	16
2-7	116	1856	16

**Table 3:** Classification accuracy of various classifiers on 1-0 using the artificial design feature method.

*k*-fold	*k*-NN	LDA	SVM	DT	MLP	GNB	AVG
3	0.9066	0.8703	0.9265	0.8264	0.7894	0.6966	0.836
5	0.92	0.9067	0.9533	0.83	0.8133	0.7367	0.86
10	0.9333	0.91	0.9633	0.8333	0.8567	0.7467	0.8739

**Table 4:** Classification accuracy of various classifiers on raw data 2 using the artificial design feature method.

*k*-fold	*k*-NN	LDA	SVM	DT	MLP	GNB	AVG
3	0.975	0.9776	0.98	0.95	0.9726	0.9377	0.9655
5	0. 9725	0.9775	0. 9775	0. 9475	0. 98	0.96	0.9692
10	0.975	0.9775	0.975	0.955	0.98	0.955	0.9696

**Table 5:** Classification accuracy of the 5-fold classifier for datasets 1-0 to 1-7.

Dataset	*k*-NN	LAD	SVM	DT	MLP	GNB	AVG
1-0	0.92	0. 9067	0.9533	0.83	0.8133	0.7367	0.8600
1-1	0.93	0.9300	0.95	0.8067	0.84	0.7367	0.8656
1-2	0.9367	0.94	0.9567	0.8233	0.8167	0.72	0.8656
1-3	0.9233	0.91	0.9367	0.78	0.81	0.6833	0.8406
1-4	0.91	0.9033	0.9567	0.81	0.7667	0.68	0.8378
1-5	0.8833	0.8733	0.91	0.8033	0.77	0.6833	0.8206
1-6	0.8667	0.8767	0.89	0.77	0.8033	0.6767	0.8139
1-7	0.8833	0.9233	0.9267	0.8	0.78	0.6867	0.8333

**Table 6:** Classification accuracy of the 5-fold classifier for datasets 2-0 to 2-7.

Dataset	*k*-NN	LAD	SVM	DT	MLP	GNB	AVG
2-0	0.9725	0.9775	0.9775	0.9475	0.98	0.96	0.9692
2-1	0.9275	0.965	0.975	0.8825	0.9575	0.845	0.9254
2-2	0.9425	0.9675	0.975	0.9025	0.97	0.88	0.9396
2-3	0.9325	0.955	0.955	0.86	0.9475	0.8175	0.9112
2-4	0.9225	0.955	0.95	0.88	0.94	0.8175	0.9108
2-5	0.91	0.9575	0.95	0.7975	0.9225	0.75	0.8812
2-6	0.93	0.9575	0.965	0.7975	0.9425	0.8425	0.9058
2-7	0.925	0.9275	0.96	0.8625	0.92	0.855	0.9083

**Table 7:** Model categorization datasets generated by dataset 1.

*k*-fold	1-0	1-1	1-2	1-3	1-4	1-5	1-6	1-7
3	0.9832	0.9663	0.9630	0.9764	0.9697	0.9697	0.9596	0.9562
5	0.9800	0.9667	0.9667	0.9500	0.9733	0.9700	0.9700	0.9833
10	0.9700	0.9833	0.9800	0.9633	0.9867	0.9800	0.9700	0.9800

**Table 8:** Model categorization datasets generated by dataset 2.

*k*-fold	2-0	2-1	2-2	2-3	2-4	2-5	2-6	2-7
3	0.9318	0.9192	0.9040	0.9091	0.8813	0.8990	0.9015	0.9192
5	0.9325	0.9475	0.9200	0.9150	0.9275	0.9400	0.9300	0.9375
10	0.9350	0.9450	0.9100	0.9275	0.9325	0.9325	0.9250	0.9525

**Table 9:** Changes of dataset 1-0 divided by different lengths of 1 to 5 seconds.

Dataset name	Length of time (s)	Sample length	Sample size
1-0	1	174	6900
1-0	2	348	3300
1-0	3	521	2100
1-0	4	695	1500
1-0	5	868	1200
1-1	1	163	6900
1-1	2	328	3300
1-1	3	491	2100
1-1	4	655	1500
1-1	5	818	1200

## Data Availability

The first dataset comes from the dataset published by Andrzejak et al. The second dataset was collected by Boston Children's Hospital.
